The article "Animal Experiment of a Novel Neurointerventional Surgical Robotic System with Master-Slave Mode" was published in 2021. Journal: Appl Bionics Biomech.

# Animal Experiment of a Novel Neurointerventional Surgical Robotic System with Master-Slave Mode

**DOI:** 10.1155/2021/8836268

**Published:** 2021-01-28

**Authors:** Keyun Liu, Yuhua Jiang, Youxiang Li

**Affiliations:** ^1^Department of Intervention, Beijing Chaoyang Hospital, Capital Medical University, Beijing 100020, China; ^2^Department of Interventional Neuroradiology, Beijing Neurosurgical Institute and Beijing Tiantan Hospital, Capital Medical University, Beijing 100050, China

## Abstract

In order to inspect and improve the system performance of the neuro-interventional surgical robot and its effectiveness and safety in clinical applications, we conducted ten animal experiments using this robotic system. Cerebral angiography was performed on ten experimental animals, and various mechanical performance indicators, operating time, X-ray radiation dosage to the experimental animals and the experimenter, and arterial damage in the experimental animals were recorded when the robotic system completed cerebral angiography. The results show that the robotic system can successfully complete the cerebral angiography surgery, and the mechanical performance is up to standard. The operating time is almost the same as the physician's operating time. And the mean X-ray radiation dosage received by the experimental animals and experimenter was 0.893 Gy and 0.0859 mSv, respectively. There were no complications associated with damage to the vascular endothelium. The robotic system can basically complete the relevant assessment indicators, and its system performance, effectiveness, and safety in clinical applications meet the standards, basically meeting the requirements of clinical applications of neurointerventional surgery.

## 1. Introduction

Vascular disease is an important cause of human death, involving all types of arteries in the whole body, but the aorta, coronary artery, carotid artery, and cerebral artery are the main sites, so myocardial infarction and cerebral infarction become the main consequences of this vascular disease. In recent years, the incidence of cardiovascular and cerebrovascular diseases is increasing, gradually becoming the disease with the highest incidence, recurrence rate, and mortality [1, 2]. There are various treatment methods for vascular diseases, mainly divided into medical and surgical treatment. Among the various treatment methods, minimally invasive vascular interventional therapy with small trauma, fast recovery, and good healing has played an increasingly important role in the treatment of cardiovascular and cerebrovascular diseases and gradually becomes the best treatment method.

However, there are still bottlenecks that restrict the development of endovascular therapy, such as the difficulty of the operation technique, the risk of surgery caused by the low stability and precision of manual operation, radiation injury, the risk of leucopenia and cell carcinogenesis caused by radiation in the long term [3, 4], the fatigue and chronic injury of interventionalists caused by heavy protective equipment [5, 6], the difficulty in the training of vascular interventionalists, the less primary medical resources, and low level of vascular interventional practice. The vascular interventional robotic system can solve these problems very well. The robotic system can be operated with high precision and stability. It can isolate X-ray operation and avoid radiation. Meanwhile, it can be used for training by surgeons who have no prior experience in interventional surgery. A variety of robotic endovascular treatment systems are now available [7–13]. However, these systems are expensive and complex, with relatively homogeneous product positioning, and all have their own limitations.

Therefore, in collaboration with Beijing Institute of Technology, we have developed a master-slave robotic system for cardiovascular and cerebrovascular interventional surgery with catheter-guidewire cooperative operation [14–18]. The robot system is divided into two parts: the master end is located outside the operating room, and the slave end is set in the operating room. The control signal is transmitted to the slave end through the doctor's operation at the console of the master end, and the operation is completed by the slave end. There is an accurate force feedback system on the operating handle of the master end, so the operator can accurately feel the change of resistance of the catheter and guidewire from the end, which increases the sense of presence of operation. The slave end device is equipped with a catheter controller and a guidewire controller to enable the catheter and guidewire to operate in concert and has a haptic feedback system. The slave end takes the form of multiple platform connection blocks on the same trajectory, and the platform connection blocks are used to secure a catheter controller or guidewire controller to control the axial movement of the catheter and guidewire on a single trajectory. Since multiple sliders are used to run on the same track, each slider runs at the same distance. The accuracy of catheter pushing and rotation is improved, and damage to the guidewire surface is reduced; all this makes interventional procedures or angiography safer and more maneuverable. Using master-slave operation, it avoids the need for the physician to operate directly under the X-ray, solving a number of problems caused by the physician's prolonged exposure to radiation. The device can also be used for simulation and training in vascular interventional procedures.

The robotic system is capable of performing a variety of vascular interventional procedures. At present, 10 cases of performance self-assessment, partial type testing, and animal testing have been completed. Through the analysis of the experimental process and results, we have further verified the feasibility and safety of the robot for clinical application, and the robot has achieved the same surgical quality as that of manual operation. This report describes the performance and safety of the robotic system in animal studies.

## 2. Materials and Methods

### 2.1. Materials

#### 2.1.1. Experimental Animals

In this study, 10 Bama miniature pigs aged 3-4 months, weighing 15-20 kg, were provided by Fulong Tengfei Experimental Animal Base. The breeding conditions and environment met the requirements of animal experiments. The miniature experimental pigs were randomly selected from the same type of experimental pigs.

#### 2.1.2. Experimental Equipment

(1) The robot of endovascular treatment is provided by Beijing Institute of Technology, which mainly includes a master manipulator and a slave robot arm
(2) Routine surgical equipment and vascular interventional surgical equipment and supplies are provided by Beijing Tiantan Hospital, which mainly include the following equipment:
  - Puncture needles: arterial puncture needles (TERUMO, Japan)
  - Arterial sheath: 5 F femoral artery sheath (Cordis Corporation, USA)
  - Guidewire: 0.035-inch hydrophilic film guidewire (TERUMO, Japan)
  - Catheter: 5 F single-bend angiographic catheter, Y-valve (Cordis Corporation, USA)
  - Microcatheter: Exel-14 microcatheters (Boston, USA)
  - Microguidewire: 0.014-inch Transend platinum microguidewire (Boston, USA)
  - Laboratory equipment: AXIOM Artis dBA DSA contrast machine, SIEMENS
  - X-ray radiation dosimeters

#### 2.1.3. Pharmaceutical Reagents

1. Sodium pentobarbital injection powder (China Pharmaceutical Group Chemical Reagent Company)
2. Heparin sodium injection (Shanghai Pioneer Pharmaceutical Company)
3. Injectable thiopental sodium (Shanghai Xinya Pharmaceutical Co., Ltd.)
4. Injectable penicillin sodium (Shanghai Pioneer Pharmaceutical Company)
5. Gentamicin sulfate injection (Guangdong Otsuka Pharmaceutical Co., Ltd.)
6. Sodium lactate ringer injection (Guangdong Otsuka Pharmaceutical Co., Ltd.)
7. 5% dextrose injection (Shanghai Baxter Medical Supplies Co., Ltd.)
8. Saline injection (Shanghai Baxter Medical Supplies Co., Ltd.)
9. Iohexol injection (Shanghai Ansheng Pharmaceutical Co., Ltd.)
10. 4% paraformaldehyde fixative solution
11. Disposable aseptic waterproof transparent plastic cover

### 2.2. Methods

#### 2.2.1. Anesthesia

Randomly selected test pigs should be injected intramuscularly with 3% pentobarbital sodium injection, 2-3 ml at a time for about 20 minutes; the injection volume and time should be changed according to the anesthesia condition.

#### 2.2.2. Fixation

The auricular vein of pigs was selected for intravenous infusion. The experimental animals were fixed on the operating table, electrocardiographic monitoring was performed, and the inguinal area was routinely disinfected and covered with a sterile sheet.

#### 2.2.3. Observation Indicators

(1) Accuracy, effectiveness, and stability indicators

- Whether the physician's console is ergonomic and capable of providing an operating platform that is consistent with the physician's habits
- The ability of the console to monitor all aspects of catheter and guidewire operation information, catheter and guidewire forces, catheter and guidewire position, and catheter and guidewire contact with blood vessels
- Whether the operating table handle is flexible and reliable and can provide force sensory feedback to the operator, making sure the procedure is carried out based on the catheter force sensing information, and the catheter force sensing information is used to determine the status of the procedure
- When the gear clamps the guidewire, it has a good fit and will not damage the coating on the guidewire surface
- The system must maintain synchronous action with the physician's operation, while also ensuring that the catheter advances in a supple manner
- The system, when installed on the operating table, should not interfere with the operation of the equipment around the operating table and has good operability
- Under the X-ray line, the system operates the movement of the guidewire catheter in the blood vessels of experimental animals, such as forward and backward movement and rotation and blood vessel superselection, which can accurately and in real time reflect the operation of the master end
- The system can deliver the catheter to the designated blood vessel in a precise and timely manner according to the doctor's instructions

(2) Safety index

- Ensure that the slave end of the robot is disinfected before each experiment, and the robot equipment can operate normally after disinfection. Meanwhile, the robot is equipped with a disposable sterile transparent plastic cover from the slave end equipment to ensure that each experimental operation is carried out under sterile conditions
- The risk of complications from endothelial damage during cerebral angiography with this robotic system is no more than 5% [19]
- Cerebral angiography time using the robotic system is not greater than the cerebral angiography time of the neurointerventionalists from different medical centers [20, 21]
- Experimenter and experimental animals were exposed to radiation doses no higher than 0.1 mSv and 1 Gy, respectively [22]

#### 2.2.4. Experimental Procedure

(1) The team from Beijing Institute of Technology installed the sterilized robotic system in the catheterization laboratory and fixed the slave end on the operating table, operating the control platform handle to test the system for satisfactory performance. The sterilized robot is equipped with a disposable sterile plastic cover to ensure the whole experiment process is carried out in a sterile environment.  Figure 1 shows the performance

(2) The sterilized 5 F single-bend angiographic catheter and 150 cm hydrophilic film guidewire were connected to the system; operating the control platform handle to control the guidewire and catheter for forward, backward, and rotational movements, guidewire and catheter movement performance is good as shown in Figure 2

(3) The experimental Bama small pig was anesthetized and fixed on the operating bed with a bandage, and the skin was prepared at the inguinal region with a diameter of 20 cm. After the inguinal area of the experimental animals was routinely disinfected and sterile treatment towels were laid, 5% lidocaine was applied to the area 3 cm below the groin for local infiltration anesthesia. The skin was cut open, the femoral artery was separated layer by layer, dissociated for about 1 cm, punctured with a puncture needle, and 5 F arterial sheath was placed (Figure 3)

(4) Adjusting the angle of the robotic system arm so that it is consistent with the inclined level of the 5 F arterial sheath, the end of the system catheter running track is approximately 3 cm from the arterial sheath to ensure that the catheter does not fold after entering the arterial sheath, which is located between the arterial sheath and the end of the track. The catheter was connected to high-pressure heparin saline, and the tip of the catheter was placed approximately 5 cm into the arterial sheath (Figure 4)

(5) Adjusting the operating table so that the guidewire and catheter are exposed under the X-ray, the doctor controls the operation handle at the operating table to keep the position of the catheter unchanged. Advancing the guidewire about 10 cm, the guidewire is seen to have entered the right iliac artery under the X-ray, rotating the head of the guidewire to point to the right. Keeping the relative position of the guidewire and catheter unchanged, while advancing the guidewire catheter, the guidewire and catheter enter the aortic arch along the abdominal thoracic aorta. Keeping the catheter position unchanged, the guidewire superselection into the right common carotid artery was controlled. Advancing the catheter along the guidewire, a suitable working position was selected, the guidewire was withdrawn, and cerebral angiography was performed, which shows good angiogram (Figure 5). The procedure is repeated 3 times, with the control handle repeatedly advancing the catheter and guidewire from the femoral artery into the abdominal aorta and then into the aortic arch and the common carotid artery. The robotic system can enter the relevant blood vessels accurately and on time each time to complete the relevant operation process

(6) The team from Beijing Institute of Technology removed the hydrophilic film guidewire from the robotic arm and attached the sterilized microcatheter and microguidewire to the system. Operating control platform handle to control the guidewire and catheter for forward, backward, and rotary movements, guidewire and catheter movement performance is good

(7) The microcatheter and the microguidewire were inserted into the single-curved angiographic catheter. Operating the handle of the platform to control the forward, backward, and rotating motion of the microguidewire and microcatheter in the single-curved angiography catheter (Figure 6), the motion performance of the microguidewire and the microcatheter was good after entering the single-curved angiographic catheter

(8) The microguidewire, microcatheter, and single-curved angiography catheter were removed, and the experimental animals were sacrificed by bloodletting (Figure 7). Samples of femoral artery, contralateral femoral artery, and bilateral common carotid artery at the puncture site were, respectively, taken for about 1 cm and fixed in 4% paraformaldehyde reagent

(9) Removing the robotic systems, operating rooms were cleaned and disinfected

(10) Paraffin-embedded specimens were cut into 4 to 7 *μ*m thick sections, and three sections were made per specimen, HE-stained, and observed under an optical microscope

#### 2.2.5. Experimental Data Collection

The following information were recorded in detail: name of experimenter, first assistant, second assistant, instrument nurse, technician and anesthesiologist, recorder, date of surgery, start time of surgery, end time of surgery, start time of anesthesia, end time of anesthesia, number of experimental animals, experiment weight of the animal, number of experiments, experimental time, time taken to switch guidewire catheters, experimenter X-ray radiation exposure, and adverse events. Some data on experimental animals are shown in Table 1.

#### 2.2.6. Pathological Section

The following image shows a pathological section of a more severely damaged arterial wall. HE staining of the femoral artery at the site of femoral artery puncture in the first animal experiment shows a whole layer inflammatory response, endothelial cells, edema, subendothelial tissue, and fibrous hyperplasia. Red blood cells, lymphocytes, leukocytes, and lamellar fibrillar-like changes are seen in the arterial wall, suggesting thrombosis (Figure 8).

In the second animal experiment, HE staining of the artery wall of the right common carotid artery showed inflammatory proliferation of endothelial cells, infiltration of lymphocytes, and tissue cell and fibrinoid changes (Figure 9).

There were no associated complications due to endothelial injury in the ten animal studies, which is less than the risk odds of complications due to endothelial injury during human manipulation for cerebral angiography.

## 3. Results

We have conducted ten animal experiments using this endovascular therapy robotic system, and the robotic system was able to successfully complete the manipulation of the guidewire and catheter into the common carotid artery for cerebral angiography. We recorded the process and results of each experiment in detail and evaluated the system performance, effectiveness, and safety of the robot system in clinical application. The results are as follows.

(1) The system is capable of accurately and timely realizing the forward, backward, and rotational motion of a single-curved angiographic catheter and 150 cm hydrophilic film guidewire in the vasculature of experimental animals under master operation. The gear with the microguidewire and microcatheter can basically complete the forward and rotation motion in the single-curved angiography catheter. The system can achieve the following indicators:

- The maximum distance of catheter pushing is 1.2 m. The accuracy of axial position detection is not less than 0.1 mm, the maximum speed is <5 cm/s, rotation accuracy not less than 5°, maximum speed of rotation < 180°/s, and switching time less than 3 min
- The disposable sterile transparent plastic cover ensures that the operating system of the slave end is sterile during the experiment. The time of cleaning and sterilization is less than 1 h
- The time of switching catheter and guidewire is less than 3 min
- DSA equipment will not affect the robot stability
- The robot can control the catheter to enter any branch vessel with an inside diameter of >3 mm and an angle of <90° to the trunk

(2) The slave end system is capable of delivering catheters into designated vessels in experimental animals in a precise and timely manner in accordance with physician instructions

(3) The console handle provides force feedback to the operator, enabling the operation to sense the status of the catheter, guidewire, microcatheter, and microguidewire. Then, according to the feedback sensory information, proceed to the next step

(4) The master end of the robot operating system basically meets the requirements of ergonomics

(5) Ten animal cerebral angiograms were performed using this robotic system without complications related to endothelial damage to the vasculature. The average operation time of 38.8 minutes is almost the same as the time of cerebral angiography operation by the neurointerventionalists from different medical centers. The average time to switch the catheter and guidewire was 2.8 minutes. The average radiation dose of experimental animals and experimenters was 0.893 Gy and 0.0859 mSv, respectively

## 4. Discussions

With the advancement of minimally invasive interventional equipment and interventional-related technologies, vascular interventional surgery has developed rapidly. However, the accuracy and stability of manual operation cannot meet the requirements of the rapidly developing vascular interventional technology, and interventionalists have long faced the problem of X-ray radiation and the inconvenience of wearing heavy protective clothing which have limited the development of interventional vascular procedures. The vascular intervention robotic system solves these problems well. There are several interventional vascular robotic systems available, but they differ greatly in terms of design philosophy and the real-world problems they solve [23–26]. Therefore, we designed this master-slave vascular interventional robot with catheter-guidewire cooperative operation according to the actual clinical needs. The system improves the accuracy and stability of vascular interventions and frees the interventionalist from X-ray radiation.

The robotic vascular interventional surgical system has been repeatedly tested and improved on a human vascular model prior to animal testing. A number of improvements and optimizations have been made to the various performance indicators. Therefore, we conducted animal experiments to further investigate and improve the robotic system. The robotic system was investigated in terms of system performance, as well as validity and safety for clinical applications.

The mechanical specifications of the robot are the basis for all operations, and we must ensure that the mechanical performance of the robot system is not compromised in different environments. Therefore, we used this robotic system to repeatedly test the mechanical properties in the vessels of experimental animals. We ran at least three tests in different vessels in each animal. In 10 animal experiments, the speed and precision of the forward, backward, and rotation of the guidewire and catheter controlled from the slave end were continuously adjustable. Simultaneously, the catheter and guidewire can cooperate with each other and be delivered at the same time, which can precisely and appropriately realize the movement of single-curved angiography catheter and hydrophilic film guidewire in the animal's blood vessels, such as forward, backward, and rotation. Its feasibility, accuracy, and stability are up to standard. Compared with manual operation, its accuracy and stability are better, which meet the requirements of clinical vascular interventional surgery.

The effectiveness and safety of robotic systems for clinical applications are mainly focused on the sterile handling of the system, the integration with the surgical environment, and the absence of harm to the patient.

In vascular interventional surgery, the catheter needs to be continuously injected with saline solution to prevent the blood flow from forming blood clots and causing vascular embolism complications. Therefore, the slave end needs to be waterproofed. At the same time, vascular interventional procedures need to be performed in a sterile environment. So we add a disposable, sterile, waterproof, and transparent membrane to the slave end, which can not only isolate the damage of normal saline to the slave end but also achieve the effect of sterilizing.

When the slave end is fused with the surgical environment, the direction of movement of the guidewire and catheter clamped by the slave end is not the same as the direction of the arterial sheath where the femoral artery is disposed. Consistently, this problem has always plagued us. After continuous experiments and improvements, we designed a special transparent sleeve that can be connected and fixed to the arterial sheath. At the same time, we added a robot arm angle-dependent adjustment device to the slave end so that the angle of the catheter guidewire entering the arterial sheath is consistent with the angle of the arterial sheath inclination.

The safety of vascular interventional procedures is mainly due to the fact that the interventional device does not cause damage to the vessel wall, which can lead to corresponding complications. After each experiment, the femoral artery, contralateral femoral artery, and bilateral common carotid artery specimens at the puncture site were collected and pathological sections were performed. The damage to the intima of the artery was observed. In the first animal experiment, due to the thin femoral artery in the experimental animals, it was difficult to puncture, and the damage to the wall of the femoral artery was greater, which belonged to human factor interference. None of the remaining animal experiments caused damage to the vascular wall, and none of them caused relevant complications.

There are still deficiencies in our experiments and robotic system. First of all, we have only conducted ten animal experiments, and we are still a long way from the application of robotic systems in the clinic, and we need more animal experiments, including further clinical trials. Secondly, for the safety evaluation of this robotic system, we only performed the evaluation of pathological sections of the vessel wall; there was no long-term observation of the postoperative situation of experimental animals. Finally, the robot system is currently in the stage of experimental development which has not been combined with DSA equipment.

## 5. Conclusions

The robot of neuro-interventional surgical has been continuously investigated and improved though 10 animal experiments. The robot system can realize the cooperative operation of the guidewire and the catheter and has a force feedback system with good accuracy and stability. And various mechanical performance indexes basically meet the needs of vascular intervention surgery. Meanwhile, the sterilization effect, integration with the operating environment, and safety index of the improved robotic system basically reach the standard.

## Figures and Tables

**Figure 1:** The manipulator arm of the slave end.

**Figure 2:** The manipulator arm of the slave end holding the guidewire.

**Figure 3:** Prepared experimental Bama small pig.

**Figure 4:** The joint between the manipulator arm of the slave end and the femoral artery sheath.

**Figure 5:** (a, b) The images of porcine cerebral angiography, respectively.

**Figure 6:** The robot system controls the microguidewire and microcatheter movement.

**Figure 7:** Femoral artery pathology specimens from experimental animals.

**Figure 8:** Pathological section of the femoral artery in the first experimental animal.

**Figure 9:** Pathological section of the right common carotid artery in the second experimental animal.

**Table 1:** Partial experimental data.

Number	Date of operation	Animal body weight	Time of operation takes	Time of switching the guidewire catheter	Experimenter X-ray radiation dose (mSv)	X-ray radiation levels in experimental animals (Gy)	Adverse event
1	2017.06.24	18 kg	45 min	4 min	0.11	1.1	Sputum interferes with breathing, give suctioning treatment
2	2017.07.29	17 kg	40 min	3.5 min	0.1	1	Sudden cardiac arrest and resuscitation
3	2017.10.21	15 kg	40 min	2.5 min	0.085	0.86	None
4	2017.10.21	18 kg	36 min	2.5 min	0.078	0.83	None
5	2018.06.23	17 kg	37 min	2 min	0.079	0.91	None
6	2018.07.28	20 kg	35 min	2.5 min	0.086	0.88	None
7	2018.08.18	19 kg	34 min	2 min	0.084	0.87	None
8	2018.09.23	18 kg	32 min	2 min	0.082	0.85	None
9	2018.10.20	19 kg	30 min	2 min	0.079	0.83	None
10	2018.11.17	18 kg	29 min	2 min	0.076	0.80	None

## Data Availability

The data of relevant parameters of the robot system used to support the findings of this study have not been made available because the robot system is in the development stage.
